# Specific Transfection of Inflamed Brain by Macrophages: A New Therapeutic Strategy for Neurodegenerative Diseases

**DOI:** 10.1371/journal.pone.0061852

**Published:** 2013-04-19

**Authors:** Matthew J. Haney, Yuling Zhao, Emily B. Harrison, Vivek Mahajan, Shaheen Ahmed, Zhijian He, Poornima Suresh, Shawn D. Hingtgen, Natalia L. Klyachko, R. Lee Mosley, Howard E. Gendelman, Alexander V. Kabanov, Elena V. Batrakova

**Affiliations:** 1 Department of Pharmaceutical Sciences, Center for Drug Delivery and Nanomedicine, University of Nebraska Medical Center, Omaha, Nebraska, United States of America; 2 Department of Pathology and Microbiology, University of Nebraska Medical Center, Omaha, Nebraska, United States of America; 3 Department of Pharmacology and Experimental Neuroscience, Center for Neurodegenerative Disorders, University of Nebraska Medical Center, Omaha, Nebraska, United States of America; 4 Eshelman School of Pharmacy, University of North Carolina at Chapel Hill, Chapel Hill, North Carolina, United States of America; 5 Department of Chemical Enzymology, Faculty of Chemistry, M.V. Lomonosov Moscow State University, Moscow, Russia; “Mario Negri” Institute for Pharmacological Research, Italy

## Abstract

The ability to precisely upregulate genes in inflamed brain holds great therapeutic promise. Here we report a novel class of vectors, genetically modified macrophages that carry reporter and therapeutic genes to neural cells. Systemic administration of macrophages transfected *ex vivo* with a plasmid DNA (*p*DNA) encoding a potent antioxidant enzyme, catalase, produced month-long expression levels of catalase in the brain resulting in three-fold reductions in inflammation and complete neuroprotection in mouse models of Parkinson's disease (PD). This resulted in significant improvements in motor functions in PD mice. Mechanistic studies revealed that transfected macrophages secreted extracellular vesicles, exosomes, packed with catalase genetic material, *p*DNA and mRNA, active catalase, and NF-κb, a transcription factor involved in the encoded gene expression. Exosomes efficiently transfer their contents to contiguous neurons resulting in *de novo* protein synthesis in target cells. Thus, genetically modified macrophages serve as a highly efficient system for reproduction, packaging, and targeted gene and drug delivery to treat inflammatory and neurodegenerative disorders.

## Introduction

Development of new delivery systems for gene and drug transport for neurodegenerative disorders, including Parkinson's and Alzheimer's diseases (PD and AD), is greatly needed. The challenges faced are: limited blood brain barrier (BBB) permeability, inherent peripheral and brain drug toxicities, and low therapeutic indices. The pathobiology of PD and AD is linked to microglial activation and subsequent secretion of neurotoxic factors. These include reactive oxygen and nitrogen species (ROS and RNS) leading to oxidative stress [1]–[4], which affects neuronal, astrocyte, and microglia function by inducing ion transport and calcium mobilization, and activating apoptotic programs. Apoptosis and excitotoxicity are principal causes of mitochondrial-induced neuronal death [5]. Indeed, the mitochondrial respiratory chain affects oxidative phosphorylation and is responsible for ROS production. Such pathways lead to neuronal demise and underlie the pathobiology of PD and AD [6].

The lack of natural antioxidants (glutathione and superoxide dismutase) and iron in the *substantia nigra (SN)* are specifically associated with the pathobiology of PD [7]–[9]. Removing ROS and affecting mitochondria function through targeted delivery of redox enzymes could attenuate disease progression [10]. Therefore, efficient brain delivery of redox enzymes, such as catalase and superoxide dismutase, or their replicative genetic material can attenuate ROS and improve disease outcomes. Unfortunately, antioxidants when administered as therapeutic agents fail to alter the course of PD-associated neurodegeneration [11]. We posit that such failures may be a result from limited delivery of antioxidants at disease sites. Taking advantage of the neuroinflamatory process and the active egress of immunocytes from blood to sites of inflammation, we developed monocytes/macrophages as drug carrier systems for inflammatory-mediated diseases [12]–[18]. The system rests in the ability of blood borne macrophages to carry antioxidant proteins across the BBB to affected brain subregions. To preclude macrophage-mediated enzyme degradation, catalase was packaged into a block ionomer complex with a cationic block copolymer, poly(ethyleneimine)-poly(ethylene glycol) producing nanosized particles, “nanozymes”. We demonstrated that such nanozyme-loaded macrophages systemically administered into mice with brain inflammation facilitated nanozyme transport across the BBB. In addition the cell-carriers provided sustained and prolonged release of catalase suggesting a depot role for the enzyme [13]. It was demonstrated that at least a portion of macrophages loaded with nanozyme migrate from the blood away into the tissue and the tissue-associated cell-carriers slowly unload and supply the blood plasma providing sustained levels of catalase in the plasma over seven days.

Furthermore, macrophages discharged nanozyme to contiguous cells facilitating decomposition of ROS, reducing neuroinflammation, and attenuating nigrostriatal degeneration that ultimately produced potent neuroprotection in PD mice. The transfer of nanozyme from macrophages to target recipient cells is by a) partial transient fusion of cellular membranes, b) formation of macrophage bridging conduits (BCs), filopodia and lamellipodia, and 3) release of exosomes, extracellular vesicles that contain the nanozyme [18].

Exosomes are specialized membranous vesicles, that are secreted by a variety of cells, particularly cells of the immune system: dendritic cells [19], macrophages [20], B cells [21], and T cells [22]. Exosomes were initially thought to be a mechanism for removing unneeded membrane proteins from reticulocytes. Recent studies have shown that they are specialized in long-distance intercellular communications facilitating transfer of proteins [23], and functional mRNAs and microRNAs for subsequent protein expression in target cells [24], [25]. The efficient cell-to-cell transfer is accomplished by facilitated membrane interactions and fusion, expression of adhesive proteins and specific vector ligands (tetraspanins, integrins, CD11b and CD18 receptors) on the surface of exosomes [19], [26]. To shuttle their cargo, exosomes can attach by a range of surface adhesion proteins and fuse with the cell-target membrane. We demonstrated previously that incorporation of nanoformulated catalase (“nanozyme”) in exosomes altered its intracellular localization in target cells of neurovascular unit (neurons, brain microvessel endothelial cells, and astrocytes) enabling to reach different intracellular compartments such as ER, cytoplasm, and mitochondria, where ROS may be efficiently deactivated by catalase [18].

Another approach for targeted cell-mediated delivery system is using genetically-modified cell-carriers that were transfected with *p*DNA encoding a therapeutic protein. In this case, transfected cells can achieve gene delivery providing a sustained expression of the therapeutic protein in the inflamed brain. It was reported that genetically-modified cell-carriers were used for successful gene therapy of PD and AD. Thus, neurotropic factors, brain-derived neurotropic factor (BDNF) [27], [28], glial cell-line derived neurotropic factor (GDNF), or vascular endothelial growth factor (VGEF) were delivered by transfected neural stem cells (NSC) [29]–[31], or bone marrow-derived macrophages [32] for treatment of PD-related inflammation and neuronal degeneration. Furthermore, transfected NSC were also used for delivery of neurotrophic factors in AD mouse models [27], [33]–[36].

Based on our previously developed cell-mediated delivery system for nanoformulated catalase, the present work utilized genetically-modified immunocytes for targeted gene and drug delivery in PD model. In particular, RAW 264.7 macrophages were transfected with *p*DNA encoding reporter proteins (GFP, or luciferase, or tomato protein), or the therapeutic protein (catalase). The gene and protein transfer from genetically-modified macrophages, and their therapeutic effect were evaluated in *in vitro* and *in vivo* PD models. We demonstrated for the first time that systemically administered transfected macrophages release exosomes with incorporated in them DNA, mRNA, transcription factors molecules, and the encoded protein. This resulted in the sustained catalase expression and subsequent potent anti-inflammatory and neuroprotective outcomes in PD models. Two models of brain inflammation were used, intracranial (*i.c.*) injections with lipopolysaccharides (LPS) or 6-hydroxidophamine (6-OHDA). We demonstrated earlier that LPS intoxications caused higher levels of neuroinflammation, which was manifested earlier than in case of 6-OHDA injections (typically 48 hours *vs.* 21 days following the intoxication, respectively) [15]. Nevertheless, hallmarks of 6-OHDA-induced neuroinflammation reflected PD-related process better than LPS-intoxications. We did not use intraperitoneal (*i.p.*) MPTP-intoxications that is also a common model of PD. The *i.p.* MPTP injections usually cause significant inflammation in peripheral organs (liver, spleen, and kidneys) that redirects considerable portion of macrophages from brain to these peripheral organs. Thus, *i.c.* intoxications with 6-OHDA and LPS are the most appropriate PD models for cell-mediated drug delivery evaluations. Overall, cell-mediated drug delivery is a promising strategy for targeted transport of therapeutic genes and drugs, which could provide a missing link for translational gene therapy of inflammatory and neurodegenerative disorders.

## Materials and Methods

### Plasmids

The gWIZ™ high expression vectors encoding the reporter genes luciferase (gWIZ™Luc) and green fluorescent protein (GFP) (gWIZ™GFP) both under control of an optimized human cytomegalovirus (CMV) promoter followed by intron A from the CMV immediate-early (IE) gene were used throughout the study (Gene Therapy Systems, San Diego, CA). The expression vector encoding tomato protein reporter gene was purchased from Clonetech Laboratories Inc. (Mountain View, CA). Human catalase *p*DNA ORF clone (NM_001752) was provided by OriGene (Rockville, MD). All plasmids are expanded in DH5α *e.coli* and isolated using Qiagen endotoxin-free plasmid Giga-prep kits (Qiagen, Valencia, CA) according to the protocol.

### Reagents

GenePORTER 30000 transfection agent was purchased from AMS Biotechnology, England). LPS, 6-OHDA, and Triton X-100 were obtained from Sigma-Aldrich (St. Louis, MO, USA). Alexa Fluor-678-conjugated anti-CD11b was purchased from BD Biosciences (San Diego, CA). Rabbit polyclonal anti-GFP antibodies (A6455), secondary chicken anti-rabbit HRP-conjugated antibodies (A829), and antibodies to human catalase (A16772-100) were obtained from Abcam (Cambridge, MA). Anti-NeuN Antibodies were purchased from EMD Millipore, (Billerica, MA). CD63 and NFκB P65 monoclonal antibodies were obtained from Santa Cruz Biotechnology (Santa Cruz, CA). A luminescent substrate, D-Luciferase, was purchased in Caliper Life Sciences (Hopkinton, MA). A nucleic acid stain, YOYO-1 iodide (491/509), was obtained from Invitrogen (Carlsbad, CA).

### Cells

A mouse macrophage cell line (RAW 264.7) was purchased from ATCC (cat # TIB-71), and cultured in Dulbecco's Modified Eagle's Media (DMEM) (Invitrogen, Carlsbad, CA, USA) supplemented with 10% FBS. Mouse catecholaminergic Cath.A neurons were purchased from American Type Culture Collection (American Type Culture Collection, ATCC, Manassas, VA, USA), and cultured in RPMI-1640 medium supplemented with 8% normal horse serum (NHS), 4% fetal bovine serum (FBS), and 1% penicillin-streptomycin. Cath.A neurons were differentiated by adding 1 mM of N6,2′-O-dibutyryladenosine 3′,5′-cyclic monophosphate sodium salt (dbcAMP, St. Louis, MO, USA) [37].

### Animals

This study was carried out in strict accordance with the recommendations in the Guide for the Care and Use of Laboratory Animals of the National Institutes of Health. The protocol was approved by the Committee on the Ethics of Animal Experiments of the University of Nebraska Medical Center (Permit Number: 05-087-12). All surgery was performed under sodium pentobarbital anesthesia, and all efforts were made to minimize suffering. Balb/c male mice (Charles River Laboratories, USA) eight weeks of age were used in the *in vivo* IVIS experiments to reduce fluorescence quenching by colored skin and fur. The animals were kept five per cage with an air filter cover under light- (12-hours light/dark cycle) and temperature-controlled (22±1°C) environment. All manipulations with the animals were performed under a sterilized laminar hood. Food and water were given ad libitum.

### Transfection of Macrophages: Protein Expression and Release

RAW 264.7 macrophages were incubated with a mixture of 2 µg/ml GFP, or catalase, or luciferase, or tomato protein *p*DNA and GenePORTER 3000 for four hours. Following incubation, the cells were washed with PBS, cultured for various time points (up to 21 days) in complete media with 20% FBS, and then GFP expression was accounted by fluorescence activated cell sorting. Next, the same conditions were used for macrophages transfection with catalase, or luciferase, or tomato protein *p*DNA under the control of CMV promoter.

For measures of the overexpressed protein release, culture media from transfected macrophages was collected at various time points, and assessed for amount of fluorescence for GFP-transfected macrophages (Shimadzu RF5000 fluorescent spectrophotometer; λ_ex_ = 488 nm, λ_em_ = 501 nm), or catalase enzymatic activity in case of transfection with catalase *p*DNA using Amplex Red assay as described previously [12]. Briefly, media samples from transfected macrophages were supplemented with Amplex Red Dye stock solution (10 U/mL HRP, 10 mM Ampex Red) for 30 minute, and ROS content was measured by fluorescence at λ_ex_ = 563 nm, λ_em_ = 587 nm according to the manufacturer's specifications. Amount of the expressed enzyme was normalized for protein content and expressed in U of catalase per mg of the protein as means ± SEM (*N* = 4). To exclude the possibility that cell death explains the release of catalase and GFP, percentage of live macrophages on the fourth day after transfection was accounted by FACS. For this purpose, transfected cells were collected, washed, stained with Alexa 488 LIVE/DEAD dye according to manufacturer's protocol, and the amount of accumulated dye was assessed (*N* = 4). The mean +/− standard deviation was less than 10%.

### Isolation of Exosomes

RAW 264.7 macrophages grown on 75T flasks (20×10^6^ cells/flask) were transfected with GFP, catalase, or tomato protein *p*DNA as described above, washed three times with PBS, and fresh media was added to the cells. Following 48 hours, cellular media was collected, filtered through 20 µM filter to eliminate cellular debris, and exosomes were isolated using Exoquick Exosome Precipitation Solution (System Biosciences, Mountain View, CA). The obtained exosomal fraction was re-suspended in PBS (500 µl, 1 mg/ml total protein), and evaluated for protein and genetic material content. In separate experiments, exosomes isolated from tomato protein-transfected macrophages were added to Cath.A neurons and dynamics of *p*DNA accumulation and the encoded protein expression in target cells were visualized by confocal microscopy.

### Atomic Force Microscopy (AFM)

Exosomes from catalase-transfected or non-transfected macrophages were isolated, and the obtained exosomal fraction at total protein 1 mg/ml was diluted 100 times in PBS. A drop of the sample was placed on positively charged mica treated with 1-(3-aminopropyl) silatrane (APS) [38] for 2 minutes, washed with deionized water, and dried under an argon flow. The AFM imaging was operated as described [17]. Image processing and the cross-section analysis were performed using Femtoscan (Advanced Technologies Center, Moscow, Russia). The height of the particles and their diameters measured at half-maximal height were obtained from the cross-section analysis. The volume was approximated by a hemisphere using the equation [39]. A standard t-test was performed for the size comparison of exosomes released from catalase-transfected and non-transfected macrophages.

### Western Blot Analysis

Western blot technique was applied to examine protein content of exosomes secreted from GFP- or empty vector-transfected RAW 264.7 macrophages, in particular, the presence of GFP and transcription factor, NF-κB. Protein concentrations were determined using NanoDrop 2000 (Nano Drop Products, Wilmington, DE). Primary rabbit polyclonal antibodies to GFAP were used at 1∶1,000 dilution. Secondary chicken anti-rabbit HRP-conjugated antibodies were used in 1∶4,000 dilution. NF-κB P65 monoclonal antibodies were used at 1∶50,000 dilution. Specific protein bands were visualized by Immobilon Western Chemiluminescent HRP Substrate kit (Millipore, Billerica, MA), and quantitated by densitometry (Bio-Rad Laboratories, Hercules, CA) [12]. To correct for loading differences in exosomal fractions, the levels of proteins were normalized to CD63 that is constitutively expressed in exosomes.

### PCR and RT-PCR Analyses

#### cDNA synthesis

Exosomes were diluted to 1 ug/µL of protein, lysed, treated with DNase and reverse transcribed using SuperScript™ III CellsDirect cDNA Synthesis System according to manufacturer's protocol. For DNA samples exosomes were lysed and treated with RNase to prepare them for PCR.

#### Polymerase Chain Reaction

PCR was performed using GFP primers (the forward sequence was 5-TCTGGGACACAAATTGGAATACAACT-3 and reverse sequence was CGGGTCTTGAAGTTCACTTTGATTC-3) using Platinum® *Taq* DNA Polymerase (Invitrogen). Final concentrations of reagents were as follows: 1× PCR buffer, 0.2 mM dNTP mixture, 1.5 mM MgCl_2_ 0.2 µM forward primer, 0.2 µM reverse primer and 2 U DNA polymererase in distilled water. 4% cDNA or RNase treated lysate (see above) was added. The reaction mixture was incubated in a thermocycler for 30 seconds at 94°C, then 35 cycles of denaturing (94° for 15–30 sec), annealing (59°C for 30 sec), and extention (72°C for 1 min) were performed. DNA was subjected to agarose gel electrophoresis (1% agarose at 60 V for 90 min) and subsequent ethidium bromide staining (.5 ug/mL Ethidium bromide in 1× TAE), and imaged with Bio-Rad Gel Doc™ instrument.

#### Real Time PCR

40 µL DEPC treated water was used to dilute cDNA and DNA obtained as described above. 3 µL of this dilution was analyzed by real-time PCR. The real-time PCR reaction was carried out using TaqMan Gene Expression Master Mix and Expression Assays (Mouse GAPDH (The forward primer was 5-TCACTGGCATGGCCTTCC-3, the reverse sequence was 5-GGCGGCACGTCAGATCC-3, and the TAMRA probe sequence was 5-TTCCTACCCCCAATGTGTCCGTCG-3 ) and custom eGFP primers (ABI Assay ID:AIWR2DN)) using manufacturer protocols on an ABI 7700 Sequence Detector System (Applied Biosystems). Results were analyzed using the ΔΔCt method.

### Production of a Lentiviral Vector (LV)

Lentiviral vectors encoding a fusion between GFP and firefly luciferase (FLuc) were created by PCR amplifying the cDNA sequences for GFP and FLuc from pEGFP (Clontech) and pcDNA-Luciferase (Addgene) with restriction enzyme sequences that were engineered into the primers. To create the final constructs, GFP was digested with *BamHI/EcoV* and FLuc was digested with *EcoV/XhoI*. The digested fragments were ligated into the *BamHI/XhoI* digested pTK402 LV transfer vector (a kind gift from Dr. Tal Kafri, The University of North Carolina at Chapel Hill). LV-GFPFLuc viral vectors were packaged in 293T by transient transfection using the psPAX2 and pMD2.G (Addgene) packaging plasmids and following previously described protocols [40].

### Confocal Microscopy Studies

GFP expression in RAW 264.7 macrophages was visualized by a confocal fluorescence microscopic system ACAS-570 (Meridian Instruments, Okimos, MI) with argon ion laser (excitation wavelength, 488 nm) and corresponding filter set. Digital images were obtained using the CCD camera (Photometrics) and Adobe Photoshop software. To visualize catalase expression, transfected with catalase *p*DNA macrophages were fixed with 4% paraformaldehyde (PFA) for 15 min, treated with 0.4% Triton for 4 min, and then stained with primary mouse antibodies to human catalase, and Alexa 488-conjugated secondary goat anti mouse antibodies (1∶200 Dilution, Invitrogen, Carlsbad, CA, USA). Non-specific interactions were blocked with 3% BSA for 30 min prior the staining with antibodies.

To examine accumulation of exosomes secreted from macrophages in neuronal cells, RAW 264.7 macrophages (20×10^6^ cells/flask) were cultured for three days in DMEM supplemented with 10% FBS, and then concomitant media was collected, exosomes were isolated with Exoquick Exosome Kit according to manufacturer's protocol, and labeled with lipophilic fluorescent dye, 3,3′-dilinoleyl-oxacarbocyanine perchlorate (DIO) [18]. Then, Cath.A neurons grown on chamber slides (1×10^5^ cells/chamber) [41] were supplemented with the DIO-labeled exosomes (1 mg of total protein/100 µl) and incubated for another 24 hours. Neurons were stained with Anti-NeuN Antibodies (blue) prior to the imaging.

To visualize genetic material and the encoded protein transfer from exosomes to neurons, *p*DNA encoded tomato protein was labeled with a fluorescent dye YOYO-1 (green) prior to macrophages transfection. Then, RAW 264.7 macrophages were transfected with YOYO-1 labeled *p*DNA encoded tomato protein, and cultured in DMEM media. To visualize genetic material transfer from exosomes to neurons, the media from the tomato protein-transfected macrophages was collected, the exosomes (0.5 mg/ml) were isolated and added to Cath.A neurons grown on chamber slides (1×10^5^ cells/chamber). Confocal images of the neurons accumulating YOYO-labeled DNA (green) and expressing tomato protein (red) were taken at different times with corresponding laser and filter sets. Neurons were fixed and stained with Anti-NeuN Antibodies (blue) prior to the imaging.

To study macrophage-mediated gene transfer *in vivo*, mice with brain inflammation induced were *i.v.* injected with GFP-transfected macrophages (5×10^6^ cells/mouse in 100 µl PBS) on day four after transfection. In the control experiment, mice with brain inflammation were *i.v.* injected with LV-GFPFLuc virus (2×10^4^ particles/100 µl/mouse). One and five days later, animals were sacrificed and perfused as described [15], main organs (brain, liver, spleen, and lymph nodes) were removed, washed, post-fixed in 10% phosphate-buffered paraformaldehyde, and evaluated by confocal microscopy. Healthy mice (without brain inflammation) were used as controls.

### Fluorescence Activated Cell Sorting (FACS)

Number of GFP-transfected macrophages and the expression levels (in relative fluorescent units (RFU) were assessed by FACS. Typically, RAW 264.7 macrophages transfected with GFP *p*DNA/GenePORTER 3000 reagent were cultured in DMEM complete media for various times, then the cells were detached, collected and the amount of the expressed GFP was accounted by FACS.

To evaluate kinetics of GFP transfer from the transfected macrophages to Cath.A neurons, GFP-transfected RAW 264.7 macrophages (1×10^6^ cells/sample) were cultured for four days in DMEM media supplemented with 20% FBS, and then added to Cath.A neurons (1×10^6^ cells/sample, 1∶1 ratio). The co-cultured cell mixture was collected at different time points and the amount of GFP in macrophages and neurons was assessed by FACS. To distinguish between the cell types, macrophages were labeled with Alexa 678-conjugated antibodies to CD 11b prior to the assessment. The expression levels GFP levels were plotted *vs.* time of co-culture.

### Induction of Brain Inflammation in Mice

For 6-OHDA and LPS intoxications, mice were stereotactically injected into *substantia nigra pars compacta* (*SNpc*) with 6-OHDA solution (10 µg 6-OHDA in 0.9% NaCL with 0.02% ascorbic acid), or LPS solution (10 µg LPS in 0.9% NaCl with 0.02% ascorbic acid), respectively, flow rate of 0.1 µL/min into the striatum (AP: +0.5; L: −2.0 and DV: −3.0 mm) [15]. Three or four weeks after 6-OHDA intoxication, or 24 hours after LPS intoxication, the animals were injected *via* the intrajugular vein (*i.v.*) with GFP−, or luciferase-, or catalase-transfected macrophages (5×10^6^ cells/mouse in 100 µl PBS).

### Bioimaging and Infrared Spectroscopy (IVIS)

To reduce fluorescence quenching by fur, Balb/c mice were shaved prior to the imaging. Luciferase-transfected macrophages were *i.v.* injected on day 3 after transfection to 6-OHDA-intoxicated mice (5×10^6^ cells/mouse in 100 µl PBS) on day 21 after the intoxication. A solution of bioluminescent substrate, D-Luciferin, was injected intraperitoneally (*i.p.*) (100 µl/mouse) before the cell adoptive transfer. Healthy animals without brain inflammation were used in the control group (*N* = 4). In another neuroinflammation model, LPS-intoxicated mice were *i.v.* injected with catalase-transfected macrophages on day four after transfection. Ten minutes before imaging, each animal received an *i.p.* injection of XenoLight RediJect Inflammation probe, a chemiluminescent reagent for monitoring inflammation (Caliper, Hopkinton, MA). This probe is offered in a ready-to-use format and can be conveniently applied to study myeloperoxidase (MPO) activity of activated phagocytes. The animals were imaged at various time points (15 minutes–40 days) post-treatment as described [13]. The chemoluminescent signal was quantified by living image® 2.50 software and presented as radiance ratio of treated animal *vs.* 24 hours after LPS injection.

### Immunohistochemical and Stereological Analyses

6-OHDA-intoxicated mice were *i.v.* injected with PBS, or catalase-transfected macrophages, or macrophages transfected with empty vector (5×10^6^ cells/mouse/100 µl) 48 hours after the intoxication. Healthy non-intoxicated animals *i.c.* injected with PBS instead of 6-OHDA were used in two control groups that were *i.v.* injected with PBS or empty-transfected macrophages (*N* = 7) 48 hours after PBS *i.c.* injections. Four weeks later, animals were sacrificed, perfused; brains were removed, washed, post-fixed, and immunohistochemical analysis was performed in 30 µm thick consecutive coronal brain sections [13]. For detection of microglia activation, tissue sections were incubated with primary monoclonal rat anti-mouse anti-CD11b antibodies (1∶500 dilution), and secondary biotinylated goat anti-rat antibodies (Vector Laboratories, Burlingame, CA, 1∶200 dilution). For the assessment of neuroprotection effect, a tyrosine hydroxylase (TH) staining was used to quantitate numbers of dopaminergic neurons (DA) [42]. The total number of TH-positive DA neurons and CD11b-positive microglia cells were counted by using the optical fractionator module in StereoInvestigator software (MicroBrightField, Inc., Williston, VT) [13].

### Behavioral Tests

For the traditional constant speed rotarod test, mice were trained and tested as previously described [43] with slight modifications. 6-OHDA-intoxicated mice (*N* = 10) were *i.v.* injected with PBS, or catalase-transfected macrophages, or empty-transfected (with GFP-encoded *p*DNA) macrophages 48 hours after intoxication and the latency to fall from the rotarod was determined at three speeds (4, 5, and 7 rpm) on day 28 after intoxication. Healthy mice with PBS *i.c.* injections were used as a control [44]. For apomorphine test, the four groups of mice (*i.c.* PBS/*i.v.* PBS; *i.c.* 6-OHDA/*i.v.* PBS, *i.c.* 6-OHDA/*i.v.* catalase-transfected macrophages, and *i.c.* 6-OHDA/*i.v.* empty-transfected macrophages) were injected with apomorphine (0.05 mg/kg, *s.c.*) on day 28 after intoxication, and rotations were scored every 10 min for 90 min [45].

### Statistical Analysis

For the all experiments, data are presented as the mean ± SEM. Tests for significant differences between the groups in *in vitro* experiments investigating transfection of macrophages, as well as in *in vivo* evaluations of therapeutic effects of different drug formulations were performed using a one-way ANOVA with multiple comparisons (Fisher's pairwise comparisons) using GraphPad Prism 5.0 (GraphPad software, San Diego, CA, USA). A standard t-test was performed when only two groups were compared (for example, for size evaluation of exosomes released from transfected and non-transfected macrophages). A minimum *p* value of 0.05 was chosen as the significance level for all tests.

## Results

### Transfection of the Cell-carriers with Reporter and Therapeutic Proteins

Efficient transfection of cell-carriers is crucial for their use as drug and gene delivery vehicles. Therefore, at first, the optimal conditions for macrophage transfection (exposure time, DNA and transfection reagent ratios) were determined. Statistically significant increases in the expression of reporter green fluorescent protein (GFP), and catalase were found (**Fig. 1**). The best results were obtained, when macrophages were transfected using GenePORTER 3000 transfection agent incubated with 2 µg/ml *p*DNA encoded GFP, or catalase for four hours, and cultured in complete media with 20% FBS. Up to 40% of cells expressed GFP with maximal gene expression by day 4 was detected by FACS (**Fig. 1 A**), and confocal microscopy (**Fig. 1 C**). A sustained protein expression and prolonged release into the media for at least 21 days was detected by GFP fluorescence, or catalase enzyme activity (**Fig. 1 B**), and confirmed by confocal microscopy in catalase-transfected macrophages (**Fig. 1 D**). Important, the pick of the GFP fluorescence in macrophages at day 4 was followed by the sharp decreases in the expression levels and number of the transfected cells indicating relatively transient transfection of macrophages with GenePORTER 3000. Noteworthy, 95.7% of transfected macrophages releasing the encoded protein were alive on day four as confirmed by FACS. This excludes the possibility that the release of catalase and GFP into concomitant media could be a result of cell death.

**Figure 1:** Transfection of macrophages with GFP or catalase *p*DNA and prolonged release of the encoded protein. Raw 264.7 macrophages were incubated with 2 µg/ml GFP (**A, C**) or catalase (**B, D**) *p*DNA and 300 µl/ml Gene PORTER 3000 transfection agent for 4 hours, washed, and cultured in complete media for various times. Levels of the encoded protein and percentage of transfected macrophages were assessed by FACS (**A**), and the expressed protein (green) was visualized by confocal microscopy on day 4 (**C**), and day 21 (**D**). Up to 40% of cells expressed GFP (**A**) with the maximum at day 4 (**A, C**) and sustained expression for at least 21 days (**D**). For the release studies, macrophages grown on 24-well plates were transfected with: GFP *p*DNA (**B**, black squares) or catalase *p*DNA (**B**, white squares), then cells were washed, cultured for different times, and amount of the expressed protein was assessed by fluorescence (GFP) or catalytic activity (catalase). In consistence with the transfection levels, maximum of the encoded protein was detected in the culture media at day 4 with sustained levels up to three weeks. Levels of fluorescence and enzymatic activity in non-transfected macrophages are shown by arrow on corresponding axes and dashed lines. Statistical significance of GFP expression levels in macrophages, and GFP or catalase released from macrophages compared to untreated cell levels is shown by asterisk (*p<0.05; **p<0.005) was calculated by one-way ANOVA. Errors are mean ± SEM, *N* = 4. The bar: 20 µm.

### Biodistribution of Systemically Administered Macrophages in Mice and Transfection of the Inflamed Brain Tissues

It was reported that macrophages can carry and release their “payload” to distal sites of inflammation in various disease conditions, as reported [13], [18], [32], [46]. Thus, we demonstrated previously that injected intravenously fluorescently-labeled bone-marrow derived macrophages can cross the BBB and deliver nanoparticles with therapeutically active enzyme to the inflamed brain tissues [13]. Here, we use two *in vivo* models, characterized by ongoing brain inflammation caused by 6-OHDA or LPS intracranial injections into *substantia nigra pars compacta* (*SNpc*). First, to examine whether genetically-modified macrophages can reach the brain and deliver their payload, image visualization and infrared spectroscopy studies (IVIS) were conducted 6-OHDA intoxicated mice. Since luminescence is less quenched by bones and tissues than fluorescence, the macrophages were first transfected *ex vivo* with luciferase *p*DNA, cultured in complete media for 3 days, and then *i.v.* injected to the mice (5×10^6^ cells/100 µl) with or without brain inflammation. In this animal model, the inflammation reaches maximum around the day 21 after intoxication, therefore, this time point was also used as the day of transfected macrophages administration. The luminescent IVIS images of dorsal planes of the injected animals revealed striking differences in luciferase levels in mice with brain inflammation (**Fig. 2 A**) compared to healthy PBS-injected animals (**Fig. 2 B**). Thus, significant luminescence with maximum levels by days 3 to 5 after adoptive cell transfer was detected in the brain of 6-OHDA-intoxicated mice. In contrast, low, if any, luminescence was detected in PBS-treated animals injected with luciferase-transfected macrophages. No luminescence was detected in another control group of 6-OHDA-intoxicated animals with systemically administered empty vector-transfected macrophages (data not shown).

**Figure 2:** Transfection of brain tissues by genetically-modified macrophages in murine models of PD. Balb/C mice were *i.c.* injected into substantia nigra pars compacta, *SNpc* with 6-OHDA (**A**), or with PBS (**B**). Twenty one days after injections, mice were *i.v.* injected with luciferase-transfected macrophages. IVIS representative images from *N* = 4 mice per group demonstrate prolonged expression of luciferase in the brain (**A**), which peaked at days 3–5 after adoptive cell transfer. Stable luciferase expression levels were attained over a month, suggesting that along with the delivered luciferase, recorded luminescence may originate from the transfected brain tissues. In contrast, low, if any, luminescence was detected in the healthy animals (**B**). **I**: whole body images, **II**: images of mouse head for corresponding time. **C**: Sections of midbrain (both hemispheres), spleen, lymph nodes and liver of Balb/C mice *i.c.* injected with LPS into *SNpc*, and then *i.v.* injected GFP-transfected macrophages (24 hour following intoxication). Brain sections obtained after 24 hours after transfer (left column) show GFP-expressing macrophages in the ipsilateral hemisphere, spleen, lymph node. No fluorescence was detected in the liver, as well as in the contralateral brain hemisphere. Notably, substantial fluorescence throughout the whole brain was demonstrated five days after macrophages administration (right column) suggesting that genetically-modified macrophages transfected ipsilateral brain tissues with inflammation. The bar: 20 µm.

Furthermore, as we reported previously, macrophages that were labeled by ALEXA 780 fluorescent dye and systemically injected to 6-OHDA intoxicated mice were not detectable in the brain area after day 18 following administration [15]. In contrast, the obtained IVIS images (**Fig. 2 A**) demonstrated prolonged (over a month after adoptive transfer) luciferase expression in the inflamed brain. We speculate that in addition to transfected macrophages, luminescence may originate from the transfected brain tissues. Notably, both dorsal (**Fig. 2 A**) and ventral (**Fig. S1**) images of mice with brain inflammation revealed no luciferase expression in peripheral organs, liver, kidney, or spleen suggesting active targeting of genetically-modified macrophages specifically to the sites of inflammation.

IVIS imaging of live animals does not allow distinguishing between expressed protein in the blood stream or brain parenchyma. To eliminate this factor, tissue sections of brain and other organs of interest were prepared from mice with neuroinflammation (LPS *i.c.* injections) that were injected with GFP-transfected macrophages (5×10^6^ cells/100 µl/mouse) (**Fig. 2 C**) one and five days following macrophages transfer. The confocal images revealed significant GFP levels by day 1 post transfer in the lesioned brain hemisphere, spleen, lymph node, and low, if any, fluorescence in liver. No GFP expression was found in control (non-injected) hemisphere of the intoxicated animals. At day 5, in addition to GFP-expressing macrophages, significant fluorescence throughout the whole brain slides was detected suggesting that genetically-modified macrophages transfected brain tissues with inflammation. Healthy mice (without brain inflammation) yielded no GFP expression within the whole brain and much lesser levels in liver, spleen, and lymph nodes (**Fig. S2**). Together these data provide initial evidence that transfected macrophages achieved targeted drug delivery to inflammation sites increasing expression of the desired protein in the brain, but not in other peripheral tissues known to be sites amenable for macrophage migration.

### Catalase-transfected Macrophages Reduce Neuroinflammation in PD Mouse Models

Linkages between neuroinflammation and nigrostriatal degeneration have been reported [47]. Thus, transfection of brain tissues to express a redox enzyme, catalase, to attenuate inflammation could serve to protect dopaminergic neurons in disease [3], [4]. The ability of catalase-transfected macrophages to reduce brain inflammation was demonstrated first, by IVIS studies in BALB/c mice stereotactically injected with LPS into *SNpc*. The extent of inflammation as a chemiluminescence signal within the brain produced by Xenolight RediJect was quantified and presented as a radiance ratio of treated animals *vs.* LPS-injected mice at 24 hours after the LPS injection (**Fig. 3 A**). LPS intoxication induced 2.3-fold increase (SEM ± 0.3, *N* = 4) in brain inflammation levels in LPS-injected mice compared to the day first after intoxication (blue curve). In contrast, systemically administered catalase-transfected macrophages cased statistically significant decreases in neuroinflammation in LPS-intoxicated mice (2.1 times, SEM ± 0.03 at day 7, *N* = 4), which was sustained for over a month after LPS intoxication (red curve). The representative IVIS images indicate complete abrogation of brain inflammation at day 30 by the single *i.v.* injection of catalase-transfected macrophages (**Fig. 3 A**).

**Figure 3:** Anti-inflammatory and neuroprotective effects of catalase-transfected macrophages in PD murine models. **A**: LPS-induced encephalitis in BALB/C mice were injected *i.v.* with catalase-transfected macrophages (red curve), or PBS (blue curve). IVIS images over 40 days were taken ten minutes after intraperitoneal (*i.p.*) injection of a XenoLight RediJect probe for inflammation. The chemiluminescent signal was quantified and presented as radiance ratios of treated animal after 24 hours after LPS injection and at various times thereafter. Genetically-modified macrophages caused prolonged decreases of neuroinflammation in LPS-intoxicated mice. IVIS representative images at day 30 are shown. (**B**) and (**C**): BALB/c mice were *i.c.* injected with 6-OHDA. Forty eight hours later animals were *i.v.* injected with catalase-transfected macrophages, and 21 days later they were sacrificed, and mid-brain slides were stained for expression of **B**: CD11b, a marker for activated microglia or **C**: TH, a marker for dopaminergic neurons. Whereas 6-OHDA treatment caused significant microglia activation and neuronal loss, administration of catalase-transfected macrophages dramatically decreased oxidative stress, and increased neuronal survival. Administration of empty-vector transfected macrophages did not affect microglia activation, or number of dopaminergic neurons in in mice with brain inflammation. Statistical significance (shown by asterisk: *p*<0.05) was assessed by a standard t-test compared to mice with *i.c.* LPS injections followed by *i.v.* PBS injections (healthy controls). Values are means ± SEM (*N* = 4).

Next, potent anti-inflammatory and neuroprotective effects of catalase-transfected macrophages were demonstrated in the 6-OHDA-intoxicated mice (**Fig. 3 B, C**). *I.c.* injections of 6-OHDA up-regulated expression of CD11b by microglia within the *SNpc* as exhibited a more amoeboid morphology in 6-OHDA-treated mice compared to ramified microglia in PBS-treated mice (**Fig. 3 B** **,** **Table 1**). In contrast, treatment of 6-OHDA-intoxicated mice with catalase-transfected macrophages resulted in the decreased levels of CD11b and 65% less activated microglia cells compared with 6-OHDA-intoxicated control animals (**Fig. 3 B** **,** **Table 1**). Finally, systemic administration of catalase-transfected macrophages completely prevented neurodegeneration in 6-OHDA intoxicated mice (**Fig. 3 C** **,** **Table 1**). The numbers of TH+ neurons in *SNpc* of 6-OHDA animals treated with catalase-transfected macrophages were significantly (*p*<0.05) greater than those 6-OHDA intoxicated, and then PBS-injected animals. Noteworthy, the number of survived TH+ neurons in the ipsilateral side of 6-OHDA-intoxicated mice treated with catalase-transfected macrophages appears to be even greater (*p*<0.05) than those in the PBS-injected of control animals, which probably developed slight brain inflammation due to PBS *i.c.* injections. This signifies that catalase-transfected macrophages can efficiently reduce 6-OHDA-induced nigrostriatal inflammation and abolish subsequent neurodegeneration. No effect on microglia activation was found in control mice that were intoxicated with 6-OHDA, and then treated with empty vector-transfected macrophages. Nevertheless, these empty vector-transfected macrophages have subtle, but statistically significant neuroprotective effect in mice with *i.c.* PBS injections (**Fig. 3 B, C** **and** **Table 1**). We hypothesized that a particular subset of alternatively activated macrophages used in these studies (*i.e.* differentiated in presence of MCSF) has a regeneration effect as was also reported in [48].

**Table 1:** Effect of catalase-transfected macrophages on inflammation and neurodegeneration in mice with PD model^a^.

Treatment	CD11b+ (cells/mm^2^)		Total N of neurons^b^ ×10^3^	
	PBS	6-OHDA	PBS	6-OHDA
PBS	10.1±1.2	90.0±11 (**)^c^	6.9±1.9	2.5±0.5 (**)
Catalase-transfected macrophages	n/a	31.2±7.0 (*)	n/a	9.7±1.4 (*, ^#^)
Empty-transfected macrophages	9.8±1.0	89.0±11.1	8.2±2.1	3.2±0.7

a BALB/c mice were i.c. injected with 6-OHDA. Forty eight hours later, the animals were *i.v.* injected with various macrophage-based formulations or PBS. Control group was *i.c.* injected with PBS, and then 48 hours later *i.v.* injected with PBS.

b Total number of neurons was calculated in ipsilateral hemisphere.

c Statistical significance is shown by asterisk: *p*<0.05 (*), and *p*<0.005 (**) compared to mice with *i.c.* PBS injections followed by *i.v.* PBS injections (healthy controls); or *p*<0.05 (#),compared to mice with *i.c.* 6-OHDA injections followed by *i.v.* PBS injections (PD controls); was performed by a1+standard t-test. Errors are mean ± SEM, *N* = 7.

Finally, behavioral tests demonstrated statistically significant improvements in motor functions upon treatment with catalase-transfected macrophages (**Fig. 4**). Specifically, the loss of dopaminergic input due to the lesion of the left nigro-striatial pathway resulted in number of full-body contralateral rotations induced by a dopaminergic agent, apomorphine. In contrast, systemic administration of catalase-transfected macrophages to 6-OHDA intoxicated mice considerably (*p*<0.05) reduced number of these rotations on the seventh week following the intoxication in apomorphine test (**Fig. 4 A**). Furthermore, the motor functions were preserved by systemic administration of catalase-transfected macrophages in 6-OHDA intoxicated animals at the levels similar to those of control non-intoxicated mice, as demonstrated in rotarod test (**Fig. 4 B**). Noteworthy, no effect on motor functions was recorded upon administration of empty-transfected macrophages.

**Figure 4:** Therapeutic effect of catalase-transfected macrophages on motor functions in a PD mouse model. BALB/c mice were *i.c.* injected with 6-OHDA. Forty eight hours later, the animals were *i.v.* injected with catalase-transfected macrophages (bars with diagonal pattern) or PBS (black bars), or empty-transfected macrophages (white bars). Control group was *i.c.* injected with PBS, and then 48 hours later *i.v.* injected with PBS (grey bars). Apomorphine (**A**) and rotaroid (**B**) tests demonstrated statistically significant improvements in motor functions upon treatment with catalase-transfected macrophages. Number of rotations (**A**) was significantly decreased in 6-OHDA-intoxicated mice treated with catalase-transfected macrophages compared to non-treated PD mice. No rotations were detected in control PBS-injected mice in apomorphine test. Time spent on the rotarod (**B**) in 6-OHDA intoxicated mice treated with catalase-transfected macrophages was the same as in healthy non-intoxicated control mice on the seventh week after the intoxication. In contrast, significant decreases were observed in 6-OHDA-intoxicated mice injected with PBS. No effect on motor functions was recorded in 6-OHDA-intoxicated mice treated with empty-transfected macrophages. Statistical significance was calculated using one-way ANOVA test. Values are means ± SEM (*N* = 10), and *p*<0.05 compared with ^a^PBS, and ^b^6-OHDA.

### Cargo of Exosomes Secreted from Transfected Macrophages

The significance of these findings is further underscored by the ability of macrophages to shed small vesicles (exosomes and microvesicles) [26] which can contain RNA, proteins and even pre-loaded in such cells nanoparticles [18]. Here we evaluated whether transfected macrophages release these extracellular organelles with encapsulated *p*DNA, mRNA and protein products. From culture supernatants, we enriched for exosomes and microvesicles and assessed this fraction for the presence of the transgene DNA and RNA by PCR and RT-PCR analyses (**Fig. 5 A, B**). The results showed presence of both DNA and RNA of the encoded protein (here GFP) in exosomes released from transfected macrophages (**Fig. 5 A**). Important, the levels of the genetic material were about four orders of magnitude greater compared to the exosomes secreted from non-transfected macrophages (**Fig. 5 B**, group 1), as well as from the cells transfected with an empty vector (**Fig. 5 B**, group 2). Western blot analysis indicated that exosomes released from transfected macrophages contained 6.1 times greater levels of the expressed transgene protein (GFP) than those obtained from cells transfected with empty vector (**Fig. 5 C**). Finally, exosomes contained considerable amount of the transcription factor, NF-κB, which is particularly involved in the GFP expression under CMV promoter (**Fig. 5 D**). This indicates that exosomes represent a highly efficient packaging system that can be used for the delivery of proteins and genetic material to target cells.

**Figure 5:** Exosomes secreted from GFP-transfected macrophages contain GFP DNA, RNA, the transcription factor, and expressed protein. Exosomes from GFP-transfected cells were collected over two days and evaluated for (**A**): GFP DNA (**1**) and RNA (**2**) by PCR analysis. Exosomes secreted from macrophages transfected with empty vector were used as a control (**3**). (**B**): Levels of GFP DNA and RNA in exosomes from GFP-transfected macrophages were compared to those from empty vector-transfected macrophages (**1**), or non-transfected cells (**2**) by Real-Time PCR analysis. **C**: expression levels of GFP (30K) in exosomes from GFP-transfected cells (**1**) or empty vector-transfected macrophages (**2**) were examined by western blot and compared to the levels of CD63 (53K). Exosomes released from GFP-transfected macrophages contained four orders of magnitude more of GFP DNA and RNA compared to non-transfected macrophages or those transfected with empty vector (**A, B**); and 6.1 times greater levels of the expressed protein, GFP (**C**). Exosomes contain substantially higher levels of NF-kb, a transcription factor that involved in GFP *p*DNA expression, compared to macrophages as demonstrated by western blot (**D**). AFM images of exosomes revealed differences between: (**E**) small donut-shaped (empty) exosomes released from non-transfected macrophages, and (**F**) large spherical (likely filled with the expressed proteins and genetic material) exosomes from catalase-transfected macrophages. The bar: 200 nm.

AFM images show round morphology of isolated exosomes from non-transfected macrophages presenting an average diameter of 48.1±0.03 nm (**Fig. 5 E**). The donut-like shape is indicative of hollow vesicles with a central depression that appears upon drying in vacuum. Notably, exosomes from catalase-transfected macrophages were significantly larger (66.5±0.05 nm, *p*<0.001) compared to exosomes from non-transfected cells with a spherical shape sans central depression that may be due to packaging of the encoded protein and its genetic material (**Fig. 5 F**).

### Accumulation of Exosomes from Transfected Macrophages in Neurons

To study the exosomal transfer, exosomes isolated from macrophages concomitant media were labeled with lipophilic dye, DIO, and then Cath.A neurons were supplemented with these pre-labeled exosomes for 24 hours. Confocal images demonstrated substantial accumulation of DIO-labeled exosomes (green) in target cells (**Fig. 6 A**). Next, to visualize the gene transfer from exosomes to neurons, *p*DNA encoded tomato protein was labeled with a nucleoside stain, YOYO-1, and then RAW 264.7 macrophages were transfected with this pre-labeled *p*DNA. Confocal images of the transfected macrophages cultured in the complete media for three days revealed the nuclear accumulation of YOYO-1-labeled pDNA (green) and the expression of the encoded tomato protein (red) in cytoplasm of the genetically-modified macrophages (**Fig. 6 B**). Finally, media from the transfected macrophages was collected in day 3, and the isolated exosomal fraction was added to Cath.a neurons (**Fig. 6 C**) to visualize genetic material transfer and the expression of the encoded protein. Indeed, the neurons exposed to the macrophage-derived exosomes first accumulated the YOYO-1-labeled *p*DNA entrapped in these exosomes on day 1, and then expressed encoded red tomato protein on day 3 (**Fig. 6 C**). The quantification of the green and red fluorescence in confocal images revealed a relatively constant amount of *p*DNA and time dependent increased expression of tomato protein (**Fig. 6 C**, graph). This suggests that exosomes released from transfected-macrophages can carry transgene and subsequently transfect neurons signifying the possible use of macrophages as proxy for gene transfer into the acceptor cells.

**Figure 6:** Accumulation of exosomes secreted from macrophages in Cath.A neurons and genetic material transfer. **A**: Cath.A neurons grown on slides were fixed and stained with Anti-NeuN Antibodies (blue, left picture); exosomes were isolated from Raw 264.7 macrophages media, stained with lipophilic fluorescent dye, DIO (green), and added to Cath.A neurons for 24 hours (right picture). **B**: Raw 264.7 macrophages were transfected with fluorescently-labeled with YOYO-1 tomato protein *p*DNA (green), and then cultured in complete media. Confocal images of transfected macrophages on day 3 show incorporation of *p*DNA (green) in the nucleus and expression of tomato protein (red) in the cytoplasm. **C**: Media from macrophages transfected as described above with tomato protein *p*DNA (labeled with YOYO-1) was collected over 24 hours, and isolated exosomes were added to Cath.A neurons for various times. Then, the neurons were fixed and stained with Anti-NeuN Antibodies (blue). Confocal images of neurons incubated with exosomal fraction demonstrated relatively constant amount of YOYO-1-labeled *p*DNA (green), and increasing in time expression levels of tomato protein (red) confirmed by the quantification of green and red fluorescence on confocal images (graph). Co-localization of YOYO-1-labeled genetic material and expressed tomato protein in neurons is manifested by yellow staining. Statistical significance of tomato protein expression levels (shown by asterisk: *p*<0.05) was assessed by a standard t-test compared to day one after transfection. The bar: 20 µm.

### Kinetics of Gene Transfer from Genetically-modified Macrophages to Target Neurons

The kinetics of the gene transfer from macrophages to neurons was validated by FACS. Here RAW 264.7 macrophages were transfected with GFP *p*DNA, cultured in the complete media for three days, and then added to Cath.A neurons at 1∶1 of macrophage-neuron ratio. To distinguish between the donor (macrophages) and receiver (neurons) cells, macrophages were pre-labeled with antibodies to CD11b before the cell sorting. About 99.8% of macrophages were labeled (**Fig. 7**, Day 0). At 48 hours of the co-culture, GFP appears to be expressed exclusively in macrophages revealed as a CD11b+ population of cells (**Fig. 7**, Day 5). Over the time, GFP expression increases in neurons along with the appearance of CD11b marker in them (**Fig. 7**, Day 7) that ultimately yields one indistinguishable cell population (**Fig. 7**, Day 12). Taking into account that Cath.A neurons efficiently accumulate exosomes from transfected macrophages (**Fig. 6 A**), we suggest that neurons co-cultured with transfected macrophages acquired some of the CD11b-containig membranes of exosomes along with GFP genetic material and the expressed protein. Noteworthy, the GFP expression levels in macrophages alone sharply declined after day 4 after transfection, as shown in **Fig. 1 A**. In contrast, the co-culture of macrophages and neurons displays a delayed GFP expression profile, with the maximal expression shifted to day 8–12 (**Fig. 7**, graph). We hypothesized that at the earlier times GFP gene expression is mostly associated with the macrophages, while at later times, expression by neurons increases and macrophage expression fades. This reinforces the notion that genetic material as well as protein products from transfected macrophages can be transferred to acceptor cells, where additional protein is synthesized *de novo*. Important, 97.6% of transfected macrophages and neurons in co-cultured mixture were alive on day 12 as confirmed by FACS.

**Figure 7:** Transfection of Cath.A neurons by GFP-transfected macrophages. RAW 264.7 macrophages were transfected with GFP *p*DNA, cultured in complete media for three days, and then added to Cath.A neurons. To distinguish between the cell types, macrophages were stained with CD11b Ab (Alexa 647). GFP levels in neurons were assessed by FACS as mean fluorescence ± SEM (*N* = 4). **A**: The representative FACS plots demonstrating GFP transfer into Cath.A neurons; **B**: Quantification of GFP levels in macrophages alone (black diamonds), and in co-culture of neurons and macrophages (white squares). GFP expression levels in neurons co-cultured with transfected macrophages increased over 5–12 days. At the same time, protein expression in macrophages at days 5–12 was already diminished, suggesting that along with GFP, its genetic material (*p*DNA and RNA) was transferred from transfected macrophages into neurons, where the encoded protein (GFP) was synthesized *de novo*. Statistical significance shown by asterisk (*p*<0.05) was calculated by a one-way ANOVA. The bar: 10 µm.

Overall, these data support the importance of macrophage-based gene and catalase carriage for PD therapies. Indeed, mechanism of this cell-mediated drug delivery is not fully understood and warrants further studies.

## Discussion

PD is the fastest growing neurologic disorder in the developed world. Although much of the pathology remains unrealized, it is known to be associated with brain inflammation, microglia activation and neurotoxic activities including ROS that facilitate neuronal damage and death [1]–[4]. Thus, the need to deliver neuroprotectants, in particular, redox enzymes involved in anti-inflammatory neuroprotection, such as catalase and superoxide dismutase (SOD), to control neuroinflammation in the affected brain cannot be overstated. Several studies have shown that reduction of the oxidative stress-related damage, including ROS-scavenging, are attractive strategies if successfully delivered to the sites of inflammation within the brain [10], [49]. Unfortunately, many promising approaches fail to show benefits in humans, in part due to severe limitations imparted by the BBB, and the lack of delivery of therapeutic polypeptides to the brain [50], [51]. Utilizing the common approach to oxidative stress, we developed a novel cell-based gene and drug delivery system of antioxidants that features tissue specificity, and efficient penetration of the BBB.

We report here developing macrophages that were stably transfected with catalase *p*DNA to produce a therapeutically active enzyme that can efficiently reduce ROS and benefit neuronal survival during upregulated oxidative stress similar to that associated with PD. To accomplish this goal, first, genetically-modified macrophages should be able to reach the brain inflammatory sites in substantial quantities; therefore their migratory activity should not be compromised by the transfection. We demonstrated here that systemically administered macrophages transfected with luciferase *p*DNA reached the inflammatory site, delivering the encoded protein to the brain in PD mouse model. Interesting, maximum luciferase expression in the brain was detected on days 3 to 5 after macrophage transfer and was prolonged over a month with upregulated protein levels. Based on our previous IVIS data [13] indicating that *i.v.* injected fluorescently-labeled macrophages reach the inflamed brain sites maximum at day 5 with further their complete elimination by day 18, we hypothesized that luminescence recorded three weeks after *i.v.* administration of luciferase-transfected macrophages may originate not only from the transfected cell-carriers, but also from the secondary transfected brain tissues. Noteworthy, little, if any, luminescence was recorded in peripheral organs in mice with brain inflammation, or in the brain of healthy controls, suggesting targeted gene and drug delivery by macrophages to the inflamed brain.

Next, to eliminate possibility recording the expressed protein in the blood vessels, slides of the main organs of mice that were injected with GFP-transfected macrophages and then perfused to wash out the blood content were examined by fluorescence confocal microscopy. The confocal images of the brain slides confirmed macrophage-mediated delivery of the overexpressed protein to the *SNpc* as early as 24 hours after systemic administration. Notably, brain tissues from the ipsilateral hemisphere demonstrate significant fluorescence throughout the *SNpc* area 5 days after macrophages administration. This reinforces our hypothesis that genetically-modified macrophages secondarily transfected brain tissues.

The major question, whether catalase transfected macrophages can produce a neuroprotective effect in PD mice was divided into two parts: i) decrease of neuroinflammation, and ii) increase of dopaminergic neuron survival. The level of inflammation was evaluated using a marker for activated microglia, antibodies to CD11b. In mice, the neurotoxin 6-OHDA reproduces most of the biochemical and pathological hallmarks of PD, including specific degeneration of dopaminergic neurons that originate in the *SNpc* and enervate the striatum. The results presented in this work clearly demonstrated that, catalase-transfected macrophages show profound anti-inflammatory and neuroprotective effects in murine models of neuroinflammation and PD. Thus, systemic administration of catalase-transfected macrophages resulted in a substantial and prolonged attenuation of neuroinflammation (over 40 days) in mice with neuroinflammation. Furthermore, catalase-transfected macrophages dramatically decreased inflammation, and increased neuronal survival in 6-OHDA-intoxicated mice. Therapeutic efficacy of the catalase-transfected macrophages was confirmed by 2.9-fold reductions in microgliosis as measured by CD11b expression, and 3.9-fold increase in tyrosine hydroxylase (TH)-expressing dopaminergic (DA) neurons as measured by TH, a marker for dopaminergic neurons, compared to 6-OHDA-intoxicated mace treated with PBS. Noteworthy, the number of survived DA neurons of mice after *i.c.* 6-OHDA intoxication followed by transfected macrophages systemic administration was even greater than those in control healthy mice *i.c.* injected with PBS. The potent neuroprotective effect by catalase-transfected macrophages was further manifested in significant improvements in motor functions in the 6-OHDA mouse model.

The most remarkable finding of this study is the fact that genetically-modified macrophages released the expressed protein and its genetic material (DNA and RNA) in exosomes, specialized membranous vesicles, that may facilitate transfer of their cargo to contiguous target neurons, similarly to the previously reported macrophages pre-loaded with drug-incorporated catalase nanoparticles [18]. Exosomes and microvesicles by themselves have attracted recently a significant attention as naturally occurring nanoparticles that may provide a noninvasive and novel therapeutic approach for efficient delivery of drugs across impermeable barriers, in particular the BBB [52]–[55]. This approach allows using individualized and biocompatible therapeutic drug delivery vehicles that can pass unrecognized by the patient's immune system (because they are, in fact, a part of immunocytes) and deliver the expressed therapeutic load to the disease site. However, two main challenges when using exosomes remain: a) the efficiency of drug loading into the exosomes, and b) targeting the exosomes to a particular cell type or organ. These challenges may be resolved by using transfected cell-carriers for targeted gene and drug delivery.

Thus, we report here that DNA and RNA of the encoded protein were detected in exosomes secreted from genetically-modified macrophages by PCR and RT-PCR analyses. The data indicate four orders of magnitude increases in both DNA and RNA levels of the encoded protein in exosomes released from transfected macrophages compared to those from non-modified cells. Next, the up-regulated amount of NF-κb, a transcription factor involved in *p*DNA expression, was detected in exosomes by western blot. This may further facilitate transfection and high expression levels of the encoded protein in target cells of a neurovascular unit (neurons, astrocytes, and brain microvessel endothelial cells). In fact, confocal microphotographs confirmed transfer of fluorescently-labeled DNA to neurons from exosomes released by transfected macrophages *in vitro*. Notably, expression of the encoded protein in the neurons was increased over time, while DNA levels remain constant. This indeed is crucial for therapeutic efficacy of an antioxidant that may have greater therapeutic effect when transferred into neurons. Furthermore, additional indications of the genetic transfer from cell-carriers to target cells were revealed in differences between the kinetics of the encoded protein expression in transfected macrophages cultured alone, or in co-culture with neuronal cells. The maximum protein expression in macrophages alone occurs on day 4 after the transfection followed by sharp decreases. In contrast, neighboring neurons pick up the expression of the protein by 8–12 days after macrophage transfection, suggesting that *de novo* synthesis of protein occurs mostly in the neurons at later times.

In this study, we clearly demonstrate the ability of macrophages to deliver genetic material to the CNS suggesting this approach may represent a new and novel alterative for gene therapy. To date, the majority of gene delivery systems have relied on viral vectors, of which adenovirus (Ad), adeno-associated (AAV), virus and retrovirus/lentivirus (LV) are the most commonly used [56], [57]. In the ideal setting, viral vectors are capable of achieving robust transgene expression. However, their application has been limited by high levels of immune system activation, minimal transduction efficiency, and reliance on direct intracranial administration [58]. When delivered systemically, studies have shown that less than 1 in 100 copies of systemically administered LV are detectable in the brain [59]. This is supported by our findings which showed expression of GFP was undetectable in the brain following intravenous infusion of LV vectors (**Fig. S3**). Although certain types of AAV are more efficient at transducting the brain [60], wide variation among serotypes is observed following systemic administration [58]. In contrast, we observed macrophages are capable of effectively and efficiently delivering transgenes into the brain. As such, macrophage-based gene therapy may offer several potential advantages over traditional viral vector therapy. First, generation of macrophage-based delivery systems may increase the ease of generation. Macrophage-based systems are not reliant on cloning of transgenes into viral backbones or by viral packaging constraints that limit the size of transgenes. Secondly, viral vectors rely on specific receptors for entry and delivery of their single DNA or RNA-based transgene that can result in low or absent tranduction. With the ability to deliver DNA, as wells as exosomes carrying protein and mRNA simultaneously, macrophage-based delivery of multiple payloads in a receptor-independent manner may overcome the low transduction efficiency observed with certain viral vectors. Additionally, the simultaneous delivery of DNA, RNA, and protein by macrophages may enhance the efficacy of therapeutic proteins compare to traditional viral vectors. Lastly, one of the greatest limitations of Ad or LV vectors is robust activation of the host immune system [57]. One could envision the transplantation of autologous macrophages carrying therapeutic transgenes. Using a patient's own cells should minimize or eliminate activation of the host immune response by the drug delivery vehicle. Despite the potential advantages of macrophage delivery, there are still numerous limitations that need to be addressed. Although we did observed gene expression for greater than 3 weeks, we anticipate transgenes delivered by macrophages will not integrate into the target cell genome and therefore will only be transiently expressed. Thus, expression will not persist as long as genes delivered by AAV or LV that are capable of genome integration. Furthermore, it is unclear how the levels of gene expression by macrophage-based delivery compare to viral-based gene delivery and how this may affect therapeutic efficacy. Extensive future investigation will be required to clearly define the precise advantages and disadvantages of macrophage-based gene therapy compared to established viral vector technology; however the results of this study clearly demonstrate the potential of this new approach.

Overall, these studies indicate that genetically-modified macrophages serve as a new type of vector for gene transfer. They implement more than only inert carrier functions by being mini-factories for multiplication, packaging, and targeted gene and drug delivery to the inflammation site. Taking into account that exosomes from macrophages may efficiently adhere to neurons due to the presence of various adhesive glycoproteins [19], [61], [62], fuse to their membranes and deliver their content [18], we hypothesized that genetic material was shuttled into neurons by this mechanism resulting in fundamental effect on neuronal survival during oxidative stress in murine models of PD.

We cannot discern at this point the main mechanism of the neuroprotective effects produced by systemically administered catalase-transfected macrophages. First, these cells may cross the BBB and deliver catalase and its genetic material to the inflamed brain (**Fig. 8, Pathway I**). Second, catalase transfected macrophages may release at least a portion of exosomes with catalase and catalase genetic material in the blood stream and then these extracellular vesicles reaches CNS independently of cell-carriers (**Fig. 8, Pathway II**). Another possibility is that exosomes released from macrophages in the peripheral organs (liver, spleen, etc.) or blood stream are taken by host circulating monocytes, residential macrophages, T cells, *etc.*, which deliver exosomes with their cargo to *SNpc* by the same route as transfected macrophages shown in these studies (**Fig. 8, Pathway III**). Indeed, further mechanistic studies are necessary to understand the role of the cell-carriers and their exosomes in the encoded protein and gene transfer from macrophages to neurons. We anticipate that this system can be used for active targeted gene and drug delivery and has a potential for clinical translation.

**Figure 8:** A pictorial scheme for cell-based gene and drug delivery. Three possible ways of therapeutic effects of catalase-transfected macrophages in PD mouse model: ***Pathway I***: macrophages transfected with catalase encoding pDNA cross the BBB and release catalase and its genetic material in SNpc; ***Pathway II***: catalase and its genetic material are released from transfected macrophages in exosomes to the blood stream and bypass the BBB independently of the cell-carriers; ***Pathway III***: gene and drug-incorporating exosomes released in the periphegral organs (liver, spleen, *etc.*) or in the blood are taken by residential macrophages, monocytes, T-cells, or dendritic cells suppressing peripheral leukocyte activation that may result in decrease of inflammation in the brain.

## Supporting Information

Figure S1 **Biodistribution of expressed Luciferase in mice with brain inflammation by IVIS.** Balb/C mice were *i.c.* injected with 6-OHDA (0.5 mg/kg) into the substantia nigra pars compacta, *SNpc*. In parallel, RAW 264.7 macrophages were transfected with luciferase *p*DNA formulated with GenePorter 3000 transfection agent, cultured in complete media for three days, and then administered through *i.v.* (5×10^6^ cells/100 µl) into the mice with brain inflammation following 21 days after 6-OHDA administration (**A**). Healthy mice were used as controls (**B**). Representative images from *N* = 4 mice per group (ventral planes) taken at various time points revealed no luminescence in the brain in both mice with brain inflammation as well as healthy animals. No luminescence was detected in peritoneal area, liver, or spleen in mice with brain inflammation.
(DOCX)

Figure S2 **Tracking of GFP-transfected Macrophages in healthy mice.** RAW 264.7 macrophages were transfected with GFP *p*DNA formulated with GenePorter 3000 transfection agent, cultured in complete media for 3 days, and then administered through intrajugular vein (5×10^6^ cells/100 µl/mouse) into the mice with brain inflammation following 24 hours after LPS administration. 24 hours later mice were sacrificed and perfused with PBS and 4% PFA. Brain, spleen, and lymph nodes were frozen; tissue specimens were sectioned with a cryostate (10 µm thick) and examined by confocal microscopy (60× magnification). Representative images from *N* = 4 animals demonstrate low, but detectable amounts of BMM in the liver (**B**), spleen (**C**), and lymph node (D). No macrophages were found in the healthy brain (**A**). The bar: 20 µm.
(DOCX)

Figure S3 **Tracking of LV-GFPFLuc virus in mice with brain inflammation.** BALB/c mice were *i.c.* injected with LPS into *SN* as described in Materials and Methods. Twenty four hours later, the animals were *i.v.* injected with LV-GFPFLuc virus (2×10^4^ particles/100 µl/mouse). One day (**A**) and 5 days (**B**) later mice were sacrificed, and perfused with PBS and 4% PFA. Brains were frozen, sectioned with a cryostate (10 µm thick), and examined by confocal microscopy (60× magnification). Representative images from *N* = 4 animals detected no fluorescence in the brain indicating that LV-GFPFLuc virus particles were not able to penetrate the BBB and deliver GFP genetic material. The bar: 20 µm.
(DOCX)
